# Implementation of Personalized Scenic Spot Recommendation Algorithm Based on Generalized Regression Neural Network for 5G Smart Tourism System

**DOI:** 10.1155/2022/3704494

**Published:** 2022-05-05

**Authors:** Shuangqin Lin

**Affiliations:** School of Liming Vocational University, Quanzhou, Fujian 362000, China

## Abstract

On the basis of the analysis of the evolution dynamics and the process of smart tourism service, this paper constructs the evolutionary game model of smart tourism service and reveals the evolution mechanism of smart tourism service based on the network platform. Based on the strategic main line of “advantages,” it proposes the design ideas and overall framework of the smart tourism service model based on the network platform, including the smart tourism information interactive service model, the element collaborative service model, and the value cocreation service model. The comparison of recommendation results shows that the recommendation error of the genetically improved generalized regression neural network algorithm is reduced, and the recommendation accuracy is better than that of the unimproved generalized regression neural network algorithm. In the recommendation scenario of click-through rate recommendation, the existing recommendation models are difficult to meet the functions of memory and generalization at the same time and cannot fully mine and combine low-level features, and the model parameters of the deep learning model are difficult to learn under the high-dimensional sparse data set of the recommendation system. To solve the problem of generalization, this paper proposes a deep CTR recommendation model based on the gradient boosting tree and factorization machine. It can fully mine low-level feature information and automatically realize low-level feature combination, which can better learn model parameters on high-dimensional sparse data sets, and the recommendation results are no longer overgeneralized. In this paper, simulation experiments are carried out on the data set, and the related recommendation models are compared. The experimental results show that the model proposed in this paper achieves better results in both the AUC (area under ROC curve) evaluation index and the cross-entropy evaluation index.

## 1. Introduction

With the continuous replacement of modern information technology, the operation mode and management of the traditional tourism industry are gradually transforming to informatization, intelligence, and personalization, which fully reflects the core position of computer information technology in the development of 5G smart tourism [1]. 5G smart tourism is based on traditional tourism methods, providing an intelligent service platform for tourism and focusing on personalized user experience, combined with a new generation of computer technology to form a huge tourism service system. 5G smart tourism is based on the new generation of information technology to meet people's personalized needs for tourism products, while improving the quality and satisfaction of the tourism service industry [2]. 5G smart tourism is developed on the basis of traditional tourism services, but 5G smart tourism is not a direct extension of traditional tourism services. 5G smart tourism will provide people with a new service experience, provide a more convenient and efficient way to obtain information, and combine tourists. Based on the tourism business, combined with a new generation of computer technology, it has become a huge tourism service system for the vast number of tourists [3].

In addition to providing knowledge sharing, intelligent management, and other functions, the author believes that the purpose of smart tourism development is to provide tourists with more efficient and personalized high-quality tourism services [4]. The recommendation of personalized tourism routes is not only an important topic for the future of smart tourism but also one of the important solutions to provide users with personalized tourism services. Most of the actual implementation is still in the research stage, and the main market is the e-commerce tourism industry. Personalized recommendation based on smart travel routes is different from general recommendations in other fields and traditional travel routes [5–7]. General recommendation algorithms and systems are based on data mining to recommend some items that recommended users will like to target users. Some users in real life may feel disgusted with these meaningless recommended items. In this paper, the research on the personalized recommendation technology of tourist routes based on the change of user interest characteristics is of great significance to the commercial recommendation and promotion of tourist routes.

This paper analyzes the connotation, characteristics, participants, and service elements of smart tourism services; constructs the process model and interaction model of smart tourism services; and studies the function, structure, and development stage of the smart tourism network platform. The evolutionary game model of tourism service reveals the evolution law of smart tourism service based on network platform; using the theory of comprehensive advantages, it proposes the overall framework of smart tourism service model based on the network platform, namely, information interaction service model, element collaborative service model, and value cocreation service model. The MATLAB neural network toolbox is used to write a relatively mature generalized regression neural network recommendation algorithm program code, and the recommendation accuracy applied to the personalized scenic spot recommendation is tested. This paper proposes a deep model based on gradient boosting decision tree (GBDT) and factorization machine (FM), namely, the GAGRNN model. The model takes into account the functions of memory and generalization. Through the cascade of GBDT and FM, the low-level feature information is fully excavated, and the low-level features are automatically combined to realize the memory function of the model; the DNN module is used to generalize the features. The effective combination of GBDT, FM, and DNN suppresses the problem of overgeneralization of recommendation results from the low-order feature level; the high-dimensional sparse features are embedded into the low-dimensional dense space by introducing an embedding layer to ensure sufficient model parameters. In order to verify the rationality of the GAGRNN model, this paper conducts a simulation experiment, analyzes the influence of the main hyperparameters of the model on the results, and compares the experimental results with the commonly used CTR recommendation models. The results show that the GAGRNN model has better performance than existing models.

## 2. Related Work

Content-based recommendation is the continuation and development of traditional information filtering technology. The recommendation has nothing to do with the user's evaluation and suggestion on the item. It is only a recommendation based on the content of the item. Data mining method is used to obtain the relevant interest information of the user from the characteristics of the transaction content. In content-based recommendation, item and user are defined according to the attributes of their respective relevant features. The system understands and obtains user interests based on the characteristics of user evaluation objects and studies the matching degree between user interest data and items to be recommended. The pros and cons of the user profile model usually depend on the choice of learning method. Common methods include vector-based representation and decision tree. Content-based user profiles require historical information and behavior data of the original users in the system, and the user interest profile model will also change with changes in user interests.

Relevant scholars believe that in essence, smart tourism is a social activity that improves the tourism experience through technological means [8]. The wisdom of smart tourism lies in the perception experience, so it is necessary to take the experience as the center of the system construction and add technology to make the tourism information service personalized. The intelligentization of consumption behavior requires the co-construction of tourism resources and consumption in tourism activities. Relevant scholars have proposed to connect various participants in the consumption link of smart tourism, strengthen the standardization of business behavior, and ensure business flexibility to build a cyclic and dynamic consumption ecosystem [9, 10].

Relevant scholars have made a development interpretation from the perspective of the specific implementation needs of smart tourism and regard artificial intelligence, Internet of Things, big data, and communication networks as the main points of smart tourism system construction [11–13]. From the perspective of innovative management and improving management efficiency, relevant scholars decompose smart tourism into the construction of cloud platform, the construction of all-round perception system, and the construction of application platform as the top-level design of building smart tourism [14]. All kinds of information collected by tourist attractions are decomposed, refined, and constructed into management instructions for decision-making [15, 16].

In the field of recommender systems, people mostly only pay attention to the relationship between users and items but do not pay attention to the environmental factors [17]. However, relying solely on the binary relationship between users and items cannot generate useful recommendations in many application scenarios [18]. For example, some users prefer to listen to recommended music in the morning and evening rather than at noon; other users may want to be recommended different types of music in different moods [19]. The contextual features extracted from these environments are used to build models for different recommendation schemes, but how to optimize these different tasks is still a problem [20].

The emergence of this method has brought new ideas to the field of recommendation services. These methods build recommendation contexts for each user directly based on their behavior. Although RNNs have been successfully applied in many fields, there are still some limitations [21, 22]. First, RNNs are suitable for solving time series problems. The training time is long, and the timeliness of commercial recommender systems is an issue that must be considered. Second, RNNs can only memorize partial sequences, which are far inferior to short sequences in long sequences [23]. Once the sequence is too long to save specific behavioral information, it will lead to a drop in accuracy. According to the current research situation at home and abroad, we can know that the current recommendation service algorithms are very mature, but they are not applicable in the field of tourism; the traditional methods are not accurate in the user modeling problem, and the effect is not good [24–26]. The scalability of the algorithm is very low, and the accurate information on the Internet is not fully utilized [27].

## 3. Methods

### 3.1. Service Traffic Statistics and Load Balancing in 5G System

After determining which services are included in the application scenario to be analyzed and the parameters of each service, we first establish a two-layer model for each service in the application scenario, that is, establish a mathematical model for the session layer and grouping layer of each service. Then, the probability density function model of the data transmission rate of a single service is obtained, and the statistical result of the data rate of the service is calculated according to the model.

Network data analytics services (NWDAF) is one of the important network functions to realize network automation and can provide data analysis services for network functions. The key issues include the analysis of NWDAF based on the historical location and movement patterns of the UE, thereby helping the network to achieve more flexible mobility management. Mode users provide customized services. In addition, as mentioned above, SON is also a very important function in network slicing and can implement control and management functions in the OAM system or gNB. In this paper, NWDAF is selected for centralized mobility recommendation, and the results are reported to the AMF and the corresponding gNB. The gNB can perform functions such as access control according to the configured policy according to the analysis information. The overall signaling flow of load balancing is shown in Figure 1.

### 3.2. Smart Tourism Service Model

Tourism service providers can be further divided into tourism factor providers (including hotels, catering, transportation, and various tourism factor suppliers), tourism intermediaries (including various travel agencies and tourism service agents), platforms, and other types. In addition, tourism bureaus, industry associations, and tourism administrative departments at all levels also undertake the roles of tourism planning, development, and construction guidance and industry management. Tourists are the core of smart tourism services, tourist demand is the premise of smart tourism services, and tourism intermediaries are links and bridges, promoting the flow of tourism information and the information connection between supply and demand.

Smart tourism services include global space resources, industry-wide element supply, whole-process service value cocreation, and multidimensional and multilevel experience. Various stakeholders form complex network links in the interaction of smart tourism services. Smart tourism services have typical ecological characteristics, make full use of information technology, build a smart tourism network platform for tourists' needs, rationally allocate and effectively integrate service resources, promote tourism service innovation, and form an efficient and sustainable smart tourism service network as shown in Figure 2.

Based on the analysis of the demand for smart tourism, the service process of smart tourism is divided into five stages, namely, mapping of tourism service demand ⟶ integration of tourism service resources ⟶ formation of tourism service plan ⟶ selection and implementation of tourism service plan ⟶ tourism service evaluation and feedback. In the process of smart tourism service, information flow, factor flow, service flow, transaction flow, etc. will be formed to promote the formation of the ecological cycle of smart tourism service.

Smart tourism services take tourists' needs as the starting point, and tourism service providers such as tourism element providers and tourism intermediaries provide tourists with a whole-process tourism service plan. Every link in the smart tourism service process requires interaction, collaboration, and communication between tourists and tourism service providers.

### 3.3. Evolutionary Game Model of Smart Tourism Service

In the process of smart tourism services, tourists, tourism intermediaries, and tourism element providers are the three most important participants. Among them, tourism intermediaries play a role in promoting the dissemination and sharing of tourism information in the process of tourism services, and through cooperation with tourism element providers, they adopt diversified marketing strategies to attract all kinds of tourists and continuously expand the tourism market. In the process of smart tourism service, the network platform also assumes the functions and roles of a part of the tourism intermediary, and also acts as a tourism service integrator, becoming a key link connecting tourism intermediaries, tourism element providers, and tourists and also promoting smart tourism.

In the process of smart tourism service, when tourism intermediaries and tourism factor providers cooperate with online platforms, they all aim at maximizing their own interests to conduct smart tourism service cooperation games. At the same time, the bounded rationality of the two makes both sides imitate and improve in the cooperation with the network platform and gradually achieve the stability of cooperation through evolutionary games. There are two cooperation strategies between the two parties and the network platform to choose: simple cooperation and deep cooperation.

Simple cooperation means that the mode of cooperation between the tourism agency or tourism element provider and the online platform is fixed; there is no intention to continue to deepen cooperation, and the purpose of cooperation between the two parties is also different, while travel intermediaries or tourism factor providers hope to get more benefits from the clicks of the network platform, that is, the benefits from network effects.

In-depth cooperation means that the two parties have very strong cooperation intentions. Through diversified cooperation methods, they will continue to develop potential tourism markets and create more and wider benefits. This form of cooperation requires tourism destinations, travel agencies, network platforms, and related organizations to cooperate with each other, that is, the benefits from synergistic effects.

M represents the cooperation between tourism intermediaries and network platforms, M_1_ and M_2_ represent the deep cooperation and simple cooperation between tourism intermediaries and network platforms, D represents the cooperation between tourism factor providers and network platforms, and D_1_ and D_2_ represent tourism factor providers, respectively. UM means that the tourism intermediary adopts the income of simple cooperation with the network platform; UD means that the tourism element provider adopts the income of simple cooperation with the network platform; X means that the three parties cooperate with each other with the network platform as the core. Y represents the excess revenue share created by the deep cooperation between the tourism factor provider and the network platform and the simple cooperation between the tourism intermediary and the network platform; Z represents the deep cooperation between the tourism factor provider and the network platform and the simple cooperation between the tourism factor provider and the network platform. CM indicates the cost of in-depth cooperation with online platforms for travel agencies; CD indicates the cost of in-depth cooperation with online platforms for tourism factor providers, and the cost of simple cooperation is not considered here; *α* represents the revenue sharing ratio of tourism factor providers in in-depth cooperation with online platforms, *β* represents the revenue sharing ratio of tourism intermediaries in in-depth cooperation with online platforms, and *γ* represents online platforms proportion of revenue sharing in in-depth cooperation.

In the initial stage, it is assumed that the probability of tourism intermediaries choosing simple cooperation with online platforms is *x*, and the probability of choosing in-depth cooperation with online platforms is 1−x; the probability of tourism factor providers choosing simple cooperation with online platforms is *y*, and the probability of choosing in-depth cooperation with online platforms is 1−y.

According to the theory of evolutionary game, the expected return of tourism factor providers by in-depth cooperation and simple cooperation with online platforms is

(1) $$\begin{array}{c} u_{1\;D1}=\left(1-x\right)\left(\beta U_{D}-\alpha C_{D}+X\right)+x\left(C_{D}-\alpha Y-U_{D}\right),\\ u_{1\;D2}=\alpha xU_{D}-\left(1-\beta \right)C_{D}. \end{array}$$

The replication dynamic equation of the evolutionary game of the smart tourism service process can be obtained by the following equation:

(2) $$\begin{array}{c} F\left(y\right)=\left(M_{1}-M_{2}\right)\left(1-y\right)\left[\gamma C_{D}+C_{M}Y-\beta \left(Y-\alpha X\right)\right]. \end{array}$$

### 3.4. Generalized Regression Neural Network Algorithm

The generalized regression neural network consists of four layers, namely, the input layer, the pattern layer, the summation layer, and the output layer. The pattern layer is the radial base layer, and the neurons are radial base neurons. Like the general artificial neuron, the radial basis neuron is equivalent to a multi-input single-output nonlinear threshold device.

The general expression of the activation function is

(3) $$\begin{array}{c} R\left(n\right)=\exp\left(-bn^{2}\right). \end{array}$$

Threshold *b* is used to adjust the sensitivity of the neuron. However, the commonly used radial basis function in radial basis neurons is the Gaussian function, so the activation function of radial basis neurons can be expressed as

(4) $$\begin{array}{c} R\left(x_{n}-c_{j}\right)=\exp\left[-\frac{2\left(x_{n}-c_{j}^{T}\right){\left(x_{n}-{}_{c}^{j}\right)}^{T}}{b\sigma^{2}}\right]. \end{array}$$

In GRNN, the rules for setting some parameters of neurons in the pattern layer are specified. First, the number of neurons in this layer is equal to the number N of training samples; secondly, the center vector *c*_j_ of the *j*th mode layer neuron is the transpose vector of the *j*th input vector *x*_j_ of the training sample. Then, the output vector of the pattern layer is

(5) $$\begin{array}{c} p_{n}={\left(\begin{array}{cccc} p_{{}_{n,0}}^{T} & p_{{}_{n,1}}^{T} & \cdots & p_{{}_{n,N-1}}^{T} \end{array}\right)}^{T}, \end{array}$$

where *n* represents the *n*th training sample. The summation layer includes two types of neurons, one of which is the denominator unit, and there is only one denominator summation neuron. The denominator unit arithmetically sums the outputs of all neurons in the mode layer, the connection weight between each neuron in the mode layer and the neuron is 1, and the output is

(6) $$\begin{array}{c} S_{Tn}=\prod_{j=0}^{N-1}\left(P_{n,j}•P_{n,j+1}\right). \end{array}$$

Another type of neuron is the molecular unit, and the number of molecular summation neurons is the dimension K of the output vector of the training sample. The molecular unit performs a weighted summation on the outputs of all neurons in the pattern layer, and the connection weight *w* of this type of neurons is set. The connection weight *w*_*j*,*k*_ is the *k*th element *y*_*j*,*k*_ in the *j*th output vector in the training sample. The output of the molecular summation neuron is

(7) $$\begin{array}{c} S_{n,k}=\prod_{j=0}^{N-1}\left(P_{n,j}P_{n,j+1}w_{j+1,k}\right). \end{array}$$

### 3.5. Design of Generalized Regression Neural Network Improved by Genetic Algorithm

The genetic algorithm first generates a population, which is a group of individuals. These individuals are simulated biological individuals, that is, the object of optimization, which is another name for the smooth factor used by GRNN in this paper. Each individual is then optimized through a series of methods. In the genetic algorithm, chromosomes are represented by strings formed by encoding, and chromosomes represent possible solutions to the problem. The values at various positions on the chromosome string are the genes of a similar organism.

Coding is an important step in the design of evolutionary computing algorithms. The choice of coding scheme is largely determined by the nature and requirements of the problem and also determines the design of subsequent genetic operations. Different coding methods have a great influence on the efficiency of genetic optimization. Therefore, in order to improve the optimization efficiency, the coding must satisfy several conditions, namely completeness, soundness, nonredundancy, minimization of the coded character set, and the approximation of adjacent code points.

Fitness is a measure of how good each individual smooth factor in the population may reach or be close to the optimal solution by referring to the degree of adaptation of biological individuals to the environment. The correspondence between the smooth factor individuals and their fitness is called the fitness function. This function is used to guide the evaluation of the pros and cons of new individuals generated by genetic manipulation. How to construct fitness function is one of the core problems of genetic algorithm. The fitness function is generally single-valued and nonnegative, and the amount of calculation is small so as to meet the fitness value requirements of some selection strategies in the algorithm evolution calculation. And it needs to be able to correctly reflect the solution space distribution in the problem solution field, meet different situations under a specific problem, and have strong generality. In this paper, a GRNN is created in the fitness function, 5 adjacent samples are taken for training, and the trained network is used to recommend the target values of the 3 samples immediately after the 5 samples, and the recommended results are compared with the real value. Here, *x* is the recommended value, X is the real value, and the fitness function is

(8) $$\begin{array}{c} f\left(x\right)={\left[\prod_{i=0}^{2}{\left(X_{i}-x_{i}\right)}^{2}\right]}^{-1/2}. \end{array}$$

Selection is an operation that selects excellent individuals from the previous generation population according to the fitness of each individual in the population, eliminates inferior individuals, and is used to determine crossover or mutation individuals. The possibility of an individual's genes being passed on to the next generation depends on the size of the individual's fitness value, and the selection operation is to select individuals according to this principle. When the fitness of an individual is high, the individual is easy to be selected, and the more times it may be selected, so its genetic genotype is easily passed on to the next generation so that the population evolves towards this genotype. Therefore, the setting of the selection operator has a great influence on the evolution result. The selection operation in this paper is to make the chance of each smooth factor individual gene inherited into the next-generation population proportional to the relative fitness of the smooth factor individual. The formula for calculating relative fitness is

(9) $$\begin{array}{c} P\left(x_{i}\right)=\frac{f\left(x_{i}\right)}{\prod_{j=0}^{N-1}f\left(x_{j}\right)}, \end{array}$$

where f(*x*_i_) is the fitness value of the *i*th member in the group and N is the size of the group.

The genetic algorithm in this paper prespecifies the maximum evolutionary algebra and stops the optimization when the maximum algebra is reached. At the same time, the genetic algorithm takes into account the changes in the fitness value of successive generations of groups.

If the maximum fitness value of successive generations does not change significantly, and the average value of the fitness value of each generation tends to the maximum fitness value, then the maximum evolution generation is reached and terminated, which is considered to be effective; otherwise, the genetic operation needs to be re-executed.

## 4. Simulation Verification and Result Analysis

### 4.1. Loss Function and Evaluation Function

The experimental environment of this experiment is the Python development software Pycharm, the development environment is Python 3.6 version and TensorFlow 2.0 version, and the related software packages include TensorFlow, Keras, NumPy, and scikit-learn. The hardware environment is CPU i5-6500, the GPU uses NVIDIA GTX1080Ti, and the video memory is 6 GB.

Each sample consists of 58 features and a label of whether it is clicked. There are 24 continuous-variable domains and 35 discrete-feature domains in the features. Some of the sample eigenvalues in the data set are missing, and some feature filling needs to be done.

In terms of data preprocessing, the data are first cleaned and the missing features in the data set are filled. For the missing values of continuous features, the median filling method is used; for the missing values of discrete features, they are filled with −1, which is represented as missing categorical features.

The loss function is the target of fitting during model training. In machine learning, the loss function used in general regression models is root mean square error (RMSE). In a few ten thousandths, the use of RMSE may lead to the recommendation result tending to 0, so the cross-entropy (Logloss) is used as the loss function here. The cross-entropy loss function is equivalent to the K-L divergence, which is used to measure the difference between the recommended distribution and the true distribution, and the expression is as follows, where *y* is the true value and y' is the recommended value.

(10) $$\begin{array}{c} L\left(x,y\right)=\left(1-y\right)•\;\log\left[y^{'}\left(x\right)\right]+0.5y•\left\{1-\log\left[y\left(x\right)\right]\right\}. \end{array}$$

The evaluation index is the standard for measuring the effect of the model. Here, the cross-entropy Logloss (Logistic Loss) and AUC (area under ROC curve) are used to evaluate the model effect. Logloss is also cross-entropy, which is used to measure the recommended click rate distribution and the actual click rate distribution. The similarity is also the loss function of the model.

AUC is the area under the ROC curve. It is often used as an evaluation index for binary classification problems. It represents the probability that two samples are randomly selected, and the click rate of positive samples (clicked samples) is greater than that of negative samples (unclicked samples). AUC expression is as follows:

(11) $$\begin{array}{c} AUC=\frac{\left[rank_{sample_{i}}-\left(M-1\right)N\right]}{\left(M•N\right)}. \end{array}$$

Among them, *sample*_*i*_ represents the *i*th sample, *rank*_*samplei*_ represents the position of the *i*th sample sorted by the recommended click rate, *M* represents the number of positive samples, and *N* represents the number of negative samples.

### 4.2. Hyperparameter Simulation Analysis

This section investigates the effect of hyperparameters in the GAGRNN model, using a univariate approach to control the hyperparameters and observe the effect on the experimental results. The experimental results compare the Logloss value, AUC value, and model convergence time of the model, where the model convergence time is the sum of the convergence time of the pretrained GBDT module and the GAGRNN model.

The pretraining GBDT module needs to use all continuous features and some discrete features to construct a training set. The selection of discrete features should be determined according to the importance of discrete features. Here, discrete features are sorted by feature importance, and a certain proportion of discrete features is selected in turn to construct GBDT training set. It can be seen from Figure 3 that the proportion of discrete features will affect the effect and convergence speed of the model. As the proportion of discrete features increases from 0 to 1, the models perform quite differently on the AUC and Logloss metrics. This is because when the input discrete features of GBDT are too few, the information of important discrete features cannot be captured, and when the input discrete features are too many, because the number of GBDT iterations and the number of output leaf nodes are fixed, and too many discrete features are added, it will bring noise to the GBDT module and reduce the model effect. In terms of convergence time, because the input features increase, the GBDT training time increases, so the convergence time is between 10 and 15 s.

The number of GBDT iterations is the number of gradient boosting trees, which is proportional to the number of leaf node features output by GBDT. It can be seen from Figure 4 that when the number of GBDT iterations increases, GBDT learns more low-level features more fully, and its leaf node features represent more accurate samples, so the GAGRNN model is more effective under the AUC and Logloss indicators. However, after increasing to a certain number, the GBDT module's representation capability reaches the bottleneck, and the model effect is not significantly improved. When the number of model iterations exceeds a certain number, the GBDT training time is longer and the output leaf features are more, so the model convergence time increases significantly and the convergence speed decreases significantly.

The number of GBDT leaf nodes refers to the number of leaf nodes in each tree, which is proportional to the number of leaf node features output by GBDT. Comparing Figures 4 and 5, we can see that the influence of the number of GBDT leaf nodes on the model is similar to that of the number of iterations on the model. When the number of leaf nodes increases, the GBDT module learns more low-order features and the model effect is improved. The number of leaf nodes also significantly affects the model convergence speed. As the number of leaf nodes increases, the model convergence speed decreases.

### 4.3. Model Comparison and Result Analysis

In terms of model comparison, the basic model of click-through rate recommendation and related combination models are selected here. Basic models include LR model, FM model, GBDT model, and DNN model. In addition, due to the characteristics of the FM-related series models (including the FM model, the DeepFM model, and the GAGRNN model), the output layer uses the sigmoid function as the output function and also uses all the first-order features, which is consistent with the LR model transformation. The LR model is then combined with the FM-related series of models.

Table 1 shows the principles and related properties of the models compared in this section. Single shallow models such as LR model, FM model, and GBDT model do not have generalization ability, and single deep model DNN also has the disadvantage of overgeneralization. In contrast, the combined model can combine the advantages of various single models, mine feature information from different model perspectives, and have a stronger ability to learn features. In the combined model, only the combination of a single shallow model is used, which has no generalization ability. Although models such as Wide&Deep and DeepFM combine shallow and deep models, taking into account the functions of memory and generalization, the learning of low-level features is still insufficient. In contrast, the GAGRNN model combines GBDT, FM, and DNN. While taking into account the memory and generalization capabilities, it also fully exploits the combination relationship between low-level features, which is theoretically more superior to other models.

Models with feature combination capabilities are better than models without feature combination capabilities, such as the FM model that learns low-order feature combinations, the GBDT model, and the DNN model that learns high-order feature combinations. In fact, in practical applications in the tourism industry, the LR model is generally added with a combination of features carefully designed by professionals to improve the effect of the LR model.

The effect of using a combined model is generally better than a single model. A single model often focuses on one aspect. For example, the LR model only focuses on first-order features, the FM model and GBDT model only focus on the combination and memory of low-order features, and DNN only focuses on high-level features.

Figures 6 and 7 show the experimental results of the above models under the Logloss evaluation metric and the AUC evaluation metric. Furthermore, Figure 8 shows the experimental results of the convergence time of the above model. The model that learns high-order and low-order features is better than the model that only learns a single feature, such as the Wide&Deep model, the DeepFM model, and the GAGRNN model. In addition, GAGRNN introduces the GBDT module, which can learn more low-level features and achieve better results. Low-order models have short convergence time and fast convergence. The convergence time of the combined model is roughly the same, but because the GBDT-related model needs to pretrain the GBDT module, the convergence time is longer and the convergence speed is slower.

## 5. Conclusion

Compared with the previous optimization methods, the optimal smoothing factor obtained by this algorithm has a smaller recommendation error, especially for the target whose recommended target value is compared with the previous time point. It is more effective when the value changes greatly. In this paper, the incremental recommendation of the data of railway freight volume and its influencing factors is adopted, rather than the direct recommendation of the data itself, and then, the recommended results are calculated to obtain the desired recommendation target value. This data processing method makes the recommendation more sensitive and makes the recommendation result closer to the real value. Aiming at the problem that the existing models cannot take into account the functions of memory and generalization, the GAGRNN model proposed in this paper uses the idea of the combined model, using the traditional machine learning module to realize the memory function of features, and using the deep learning module to realize the generalization function of features. Aiming at the problem that the parameters of the deep learning module are difficult to learn in the high-dimensional sparse data set and the recommendation results are overfitted, this paper introduces the embedding layer to embed the original high-dimensional sparse features into the low-dimensional dense feature space. The model parameters can be fully learned. In the form of a combined model, the overgeneralization of the recommendation results is suppressed from the low-order feature level. In order to verify the effectiveness of the GAGRNN model, this paper uses a large data set of the relevant competition platform for simulation experiments, studies the influence of different hyperparameters of the model, and compares the experimental performance of the model with other single models and combined models. The model achieves better experimental results on AUC and Logloss evaluation metrics.

## Figures and Tables

**Figure 1:** 5G system load balancing signaling process.

**Figure 2:** The composition of the smart tourism service network.

**Figure 3:** The effect of GBDT discrete feature scale on the model.

**Figure 4:** The effect of GBDT iterations on the model.

**Figure 5:** Influence of the number of GBDT leaf nodes on the model.

**Figure 6:** Comparison of different recommendation models Logloss.

**Figure 7:** AUC comparison of different recommendation models.

**Figure 8:** Comparison of convergence time of different recommendation models.

**Table 1:** Comparison of different recommendation models.

Model number	Model	Characteristic	Type
1	DeepFM model	Memory and generalization using FM and DNN	Combination model
2	GBDT model	Prediction based on decision tree memory of feature rules	Gradient boosted tree model
3	LR model	The simple weighting of the first-order features is nonlinearly changed to fit the target	Generalized linear model
4	GBDT + FM model	Learning GBDT leaf node features using FM	Combination model
5	LR + GBDT model	Learning GBDT leaf node features using LR	Combination model
6	FM model	Use latent vectors to characterize features and calculate second-order combined feature weights	Generalized linear model
7	Wide&Deep model	Use LR and DNN to achieve memory and generalization functions, respectively	Combination model
8	DNN model	Fit complex predictive functions using multiple layers of linear weighting and nonlinear transformations	Deep learning model
9	GBDT + DNN model	Learning GBDT leaf node features using DNN	Combination model
10	GAGRNN	Implement memory and generalization	Combination model

## Data Availability

The data used to support the findings of this study are available from the corresponding author upon request.
